The article "The Effects of Exercise Interventions on Mental Health in Chinese Older Adults" was retracted in 2023. Reasons: unreliable results or conclusions; concerns about the data; concerns about the peer review; concerns about the citations.

# The Effects of Exercise Interventions on Mental Health in Chinese Older Adults

**DOI:** 10.1155/2022/7265718

**Published:** 2022-06-30

**Authors:** Lijun Wang, Shuwei Li, Lin Wei, Bo Ren, Meng Zhao

**Affiliations:** ^1^Institute of Physical Education, Soochow University, SuZhou 215000, China; ^2^Institute of Physical Education and Health, Yulin Normal University, Yulin 537000, China; ^3^Shanwei Vocational and Technical College, Shanwei 516600, China; ^4^Key Laboratory of Competitive Sport Psychological and Physiological Regulation, Tianjin University of Sport, Tianjin 301617, China; ^5^School of Economics and Management, Shanghai University of Sport, Shanghai 200438, China

## Abstract

**Objectives:**

The aim of this meta-analysis was to comprehensively evaluate the effects of exercise interventions on mental health in Chinese older adults, according to the effects of intervention methods, intervention duration, intervention frequency, intervention time, measurement tools, and subject types.

**Methods:**

We searched CNKI, Wanfang and Technology Journal Database for randomized control trials, 15 original studies were extracted, reporting on 1509 Chinese older adults (Age: 55–79 years old). We used CMA2.0 software. After heterogeneity test, suitable random effect model was selected.

**Results:**

Physical exercise had a positive effect on mental health in Chinese older adults, combined effect [SMD = −1.25, 95% CI (−1.66, −0.84), *P* ≤ 0.001], anxiety combined effect size [SMD = −1.45, 95% CI (−2.08, −0.83), *P* ≤ 0.001], depression combined effect size [SMD = −1.02, 95% CI (−1.56, −0.48), *P* ≤ 0.001]. Significant differences in the intervention types, intervention duration, intervention frequency, intervention time, and measurement tools were found.

**Conclusion:**

Physical exercise had positive intervention effect on the mental health of the Chinese older adults, which was applicable to all older adults. Exercise rehabilitation was the more effective, and the best intervention effect on the older hypertension. Due to the high heterogeneity of this study and the limited number of included literature, more high-quality needed to be included in the subsequent studies.

## 1. Introduction

In October 2016, the Central Committee of the Communist Party of China and The State Council issued the outline of the “Healthy China 2030” plan, which mentioned “strengthening the popularization of psychological health and improving mental health literacy,” and promoting mental health into a major strategy of national development. With the advance of population aging, the health problems of the older adults are becoming increasingly prominent. As a part of healthy aging [1], mental health has become an indicator to evaluate the health status of the older adults. Mental health is a manifestation of people's good psychological quality and an important part of people's overall health [2]. Previous studies have found that physical exercise, as a means to improve the physical health of the older adults, affects the development of their mental health [3]. And developed a one-year physical exercise strategy for 180 elderly people, and found that their mental health score was significantly higher than the control group, and their anxiety and depression indicators were significantly lower [4]. Fu obtained the same result. They investigated the elderly with more than 12 years of swimming experience, and found that the mental health of the older adults with long-term exercise was significantly higher than that of their peers, anxiety and depression indicators were significantly lower, and the effect of exercise intervention was more obvious in the female older adults [5]. Meta-analysis confirmed that physical exercise also has positive effects on mental health of college students and drug addicts [6,7]. However, Zhang found that the two kinds of qigong exercises did not significantly improve the depressed mood of the older adults [8].

The high inconsistencies of these results suggest the need for systematic evaluation of existing studies based on quality control. Previous studies in English languages have discussed the mental health problems of middle-aged and older adults [9], but they only involve physical and mental exercise, without specific analysis of Chinese older adults groups. Taking part in physical exercise in the Chinese older adults, the project of obvious aboriginality, at the same time, China's elderly will help their children to look after the next generation after retirement, also stressed that “to elderly with love,” and in the countryside will also exist “left-behind elderly,” this is obviously different from life in the elderly is abroad, which has differences of pressure, and that affects mental health. Therefore, it is necessary to explore the effect of physical exercise on the mental health of the Chinese older adults. So, what is the effect of physical exercise on the mental health intervention of the Chinese older adults? What are the moderating factors? These are all to be resolved.

In this study, a sample of Chinese older adults was included in a randomized controlled experimental study, which in the way of intervention, intervention in a single time, the frequency of intervention, intervention, measuring tools, and the participants of the type on the adjustment variable, in mental health and anxiety, depression for results variables, using the meta-analysis to explore the effect of physical exercise of mental health for the Chinese older adults. In order to obtain more comprehensive and objective results, but also can integrate the research design, improve the application value of physical exercise projects.

## 2. Materials and Methods

This systematic review was conducted according to the Preferred Reporting Item for Systematic Review and Meta-Analyses (PRIMA) guidelines [10].

### 2.1. Search Strategy

We searched CNKI, Wanfang and Technology Journal Database, and the key words were mental health, mental state, psychological symptoms etc. Anxiety, anxiety symptoms, depression symptoms, and other outcome indicators; physical exercise, physical activity, exercise, and other intervention words; paired combinations of words performed by older adults subjects. In order to prevent omissions, we also search the references which obtain literature and review. The deadline is October 31, 2021.

### 2.2. Selection Criteria

The selection criteria were based on the PICOS criteria in order to define the characteristics of the included studies. Population: studies including Chinese older adults participants over 55 for age were included; Intervention: studies evaluating the effect of physical exercise were included; Comparator: studies comparing other exercise or no exercise were included; Outcomes: studies assessing mental health were included; Studies design: studies with experimental studies and any type of design (i.e., within-subject and between-subject designs) were included. One reviewer initially performed the article search, after which one reviewer screened the titles and abstracts of studies identified for potential selection by the search. Any disagreements were discussed with each other, until a consensus was achieved.

### 2.3. Methodological Quality Assessment

Studies included in the meta-analysis were further assessed using the PEDro scale. This instrument evaluates both internal and external validity, gives a score out of 10, and is a reliable scale of the methodological quality of randomized control trials. Each article was scored independently by two reviewers, and divergent scores were settled by discussion.

### 2.4. Data Extraction

Information on study details (i.e., author, year, sample size, average, standard deviation, intervention type, intervention duration, intervention frequency, intervention time, measurement tools, subject older adults types, and outcome variables) were extracted from all the included studies. If there was any missing or vague information, we contacted the original author to obtain the corresponding information. Data from included studies extracted independently by two of the reviewers and any discrepancies were solved by discussed with each other.

### 2.5. Data Analysis

Statics were calculated using CMA2.0 and IBM SPSS Statistics 21. The sample size and mean post-pre intervention score with standard deviation (SD) from intervention as well as control groups were used to calculate the standardized mean differences (SMD). To assess the heterogeneity *I*^2^ was considered, and 25%, 50%, and 75% were taken as the boundary values of low heterogeneity, medium heterogeneity, and high heterogeneity [11]. The publication bias test was performed using the Funnel Plot and Rosenthal's Classic Fail-safe N test.

## 3. Results

### 3.1. Search Results

A total of 1004 articles for potential inclusion were initially retrieved through the search. After removing duplicates, 481 articles remained for further screening of titles and abstracts. Afterward, 190 full-text articles were assessed for examination of their eligibility. Finally, 15 articles were included in the systematic review. The specific criteria for the screening process are shown in Figure 1.

### 3.2. Quality of Studies

According to the PEDro scale, the quality of the 15 included articles was evaluated. The score ranged from 5 to 8. The results are shown in Table 1. The quality of the included studies was above medium level, and the overall research quality was relatively good.

### 3.3. Study Characteristics

The study characteristics included the author (year), intervention types, intervention duration, intervention frequency, intervention time, measurement tools, subject older adults types, and outcome variable (Tables 2 and 3). According to the different types of intervention methods included in the original study, intervention types were divided as follows: traditional exercise (7: referring to the number of literature included in this meta-analysis), walk (2), dance (6), and exercise rehabilitation (2). The duration of a single intervention was divided as follows: less than 30 minutes (2), 30–60 minutes (including 30 and 60 minutes, 12), and more than 60 minutes (3). As regular exercise (more than three times per week) was used in the included literature, intervention frequency was divided as follows: 3–6 times per week (12) and 7 times per week (5). Intervention periods were divided as follows: less than 12 weeks (1), 12–16 weeks (10), and more than 16 weeks (6).

Each article was coded independently by two reviewers, and divergent conditions were settled by discussion. The coding consistency was 93.67%.

Square dance: a rhythmic dance performed spontaneously by Chinese residents in open spaces, such as squares and courtyards, for the purpose of fitness usually accompanied by loud rhythmic music. Artery-relaxed scripture: an exercise method in fitness qigong to strengthen the body and strength, its main feature is the combination of movement and stillness, internal stillness to collect the heart and breath, external movement to strengthen the muscles and bones. Fitness dance: a dance used for bodybuilding and slimming, through the movement of the whole body muscles to achieve the effect of trimming the body, beautiful lines. Five-animal exercises: a gymnastic exercise created by Hua Tuo that imitates the activities of animals (tigers, deer, bears, apes, and birds (cranes)) and has a good exercise effect on the body and the five organs. Exercise rehabilitation: the exercise method mainly includes aerobic training, resistance training, and flexibility and balance training, all of which are based on the physical condition of the elderly and adhere to the principle of gradual progress.

### 3.4. Publication Bias Assessment

The effect value of physical exercise on the mental health intervention effect of the older adults was concentrated on both sides of the total effect value (Figures 2–4). From the subjective funnel plot, it can be seen that there is no serious publication bias in the research on the effect of physical exercise on the mental health of the Chinese older adults, but it still needs to be further tested.

Physical exercise on the intervention effects of mental health, anxiety, and depression, which loss of safety factor is, respectively, 1502, 1268, and 606 (Table 4), namely, the corresponding amount of literature is needed to deny the current judgment of the effect of physical exercise on mental health in the older adults, it shows that the current outcomes are no publication bias.

Heterogeneity test (*I*^2^ = 95.03) (Table 4) and I-Squared >75% indicated high heterogeneity. It also indicated that 95.03% variation of the indicators of the effect of physical exercise on the mental health of the older adults was caused by the real difference in the effect value, and the study was also affected by intergroup errors. Therefore, the random effect model was used in this study to further explore the source of heterogeneity.

### 3.5. The Effect of Physical Exercise on Mental Health of Chinese Older Adults

A comprehensive analysis of the effect of physical exercise on the mental health of the older adults shows the combined effect of mental health [SMD = −1.25, 95% CI (−1.66, −0.84), *P*=0.000 < 0.001], the combined effect of anxiety [SMD = −1.45,95% CI (−2.08, −0.83), *P*=0.000 < 0.001], and the combined effect of depression [SMD = −1.02,95% CI (−1.56, −0.48), *P*=0.000 < 0.001] (Table 5). The results show that the total effect of physical exercise on the mental health of the older adults which intervention group is better than the control group, indicating that as long as the exercise, it will improve the mental health, anxiety, and depression of the older adults.

### 3.6. Results of Subgroup Analysis of Effect Sizes

Heterogeneity tests showed that there was high heterogeneity among studies, which may indicate a significant moderating effect. Subgroup analysis is one of the common methods to explore the source of heterogeneity. Therefore, this study further explores the source of heterogeneity and its regulatory effect by subgroup analysis. This study explored intervention types (traditional exercise, walk, dance, and exercise rehabilitation), intervention duration (less than 30 minutes, 30–60 minutes, more than 60 minutes), intervention frequency (3–6 times/week, 7 times/week), intervention time (less than 12 weeks, 12–16 weeks, more than 16 weeks), measurement tools (GDS, SAS, SCL-90, SDS, STAI, and BFS) and the subjects older adults types (healthy, female, hypertension, and rural empty nesters in rural areas)

The effect of physical exercise types on mental health (*P* < 0.001), anxiety (*P* < 0.001), and depression (*P* < 0.001) of the older adults had a positive effect. Among them, exercise rehabilitation had the greatest effect on mental health (*d* = −2.50), anxiety (*d* = −2.62), and depression (*d* = −3.77) (Table 6).

The intervention time of physical exercise on mental health (*P* < 0.001), anxiety (*P* < 0.001), and depression (*P* < 0.001) of the older adults had a positive effect. Among them, the intervention time of 12 to 16 weeks had the greatest effect on mental health (*d* = −1.46) and anxiety (*d* = −1.70), and the intervention time of more than 16 weeks had the greatest effect on depression (*d* = −1.54) (Table 9).

The physical exercise on the measurement tools of mental health of the older adults (*P* < 0.001), anxiety *P* < 0.001), and depression (*P* < 0.001) had a positive effect. Among them, the intervention effect of physical exercise measured by STAI on mental health of the older adults (*d* = −2.91), anxiety (*d* = −3.01) was relatively high, measured by SDS on depression of the older adults (*d* = −2.68) is relatively high (Table 10).

The physical exercise on the older adults types of mental health (*P* < 0.001), anxiety (*P* < 0.001), and depression (*P* < 0.001) had a positive effect. Among them, the effect of physical exercise on mental health (*d* = −4.97) and anxiety (*d* = 4.97) of hypertension was higher than that of healthy older adults, female older adults, and rural empty nesters, and the effect of physical exercise on depression of healthy older adults was higher than that of female elderly and rural empty nesters (Table 11).

## 4. Discussion

### 4.1. The Effect of Physical Exercise on Mental Health of Chinese Older Adults

Through meta-analysis, this study conducted a comprehensive quantitative analysis of 15 Chinese literature on the effect of physical exercise on the mental health of the Chinese older adults. GDS, SAS, SDS, SCL-90, STAI, and BFS scales were selected to evaluate mental health, including three indicators of mental health, anxiety, and depression.

It was showed that physical exercise had a positive impact on the mental health of the Chinese older adults, that is, physical exercise could help improve the mental health level of the Chinese older adults. Compared with depression, physical exercise had the greatest effect on anxiety. Previous studies had suggested that the greatest benefits of exercise lie in the psychological domain, not in the physical domain [26]. Meta-analysis of Ma and Chen showed that the physical exercise can effectively improve the mental health of college students [27], and other studies had shown similar results, confirming that the physical exercise is a method to reduce the anxiety and depression [28–32]. This was consistent with the results of this study on the Chinese older adults. Therefore, we should pay attention to the effect of physical exercise on the mental health of the older adults, especially their anxiety. Physical exercise could improve the anxiety and depression of the older adults and then improve the individual mental health level.

### 4.2. Subgroup Analysis of Effect Sizes

Due to non-homogeneity, subgroup analysis was conducted to explore the effect of physical exercise on the mental health of the older adults, and conducted on the intervention types, intervention duration, intervention frequency, intervention time, measurement tools, and subject older adults types.

#### 4.2.1. Intervention Types

It was showed that the effect of physical exercise intervention types on mental health of the older adults had a positive effect. At present, the exercise intervention for the mental health of the older adults is still based on traditional exercise, which was related to the local exercise mode in China, it had a long history, and had been handed down to the present [32,33]. The effect of exercise rehabilitation was better than walk, dance, and traditional exercise. First of all, because of their walk's intensity was appropriate and mild, it could relieve the emotional tension caused by physical reasons in the older adults to a certain extent. Secondly, dance could increase the communication between the older adults and their peers, had more opportunities to obtain social support, and make each other find a sense of belonging and community, thus improving their mental health status [34]. Thirdly, traditional exercises, including Tai chi and qigong, could improve the emotional conditions of the older adults. For example, Tai chi can effectively regulate the emotional conditions of the older adults. The exercise program focused on “mental concentration,” focused the mind and eliminating distractions. In addition, abdominal breathing could also help regulate emotions and relieve stress [35], which was confirmed by the meta-analysis results of [36]. And Yijinjing, qigong also had the effect of pleasure. Finally, exercise rehabilitation could improve some physical conditions in a more targeted way, thus improving the mental health level of individuals and achieving antianxiety and depression effects [37]. In the future, physical exercise programs that are more suitable for the physical and mental conditions of the subjects can be developed.

#### 4.2.2. Intervention Duration, Frequency, and Time

It was showed that the duration of a single intervention of physical exercise had a positive effect on the mental health of Chinese older adults. Most studies had used intervention time of more than 30 minutes, interestingly, but the intervention effect of less than 30 minutes of exercise is higher than 30–60 minutes and more than 60 minutes. The frequency of physical exercise intervention had a positive effect on the mental health of Chinese older adults. The intervention effect of daily physical exercise was higher than 3 to 6 times a week. The intervention time of physical exercise had a positive effect on the mental health of the Chinese older adults. The intervention effect of 12 to 16 weeks of exercise was higher than that of less than 12 weeks and more than 16 weeks. They might be because of exercise in small amounts, several times a week, and in moderation is more suitable for older people, neither making them feel physically tired nor reducing their psychological benefits. Prof Ji believed that exercisers regularly exercise for 20–60 minutes each time, which was conducive to improving mood and forming a good emotional state [38]. The results of intervention dose suggest that the study of mental health intervention for the older adults was cost-effective, and the intervention time was not the longer the better. Physical activity for less than 30 minutes a day and 12 to 16 weeks had the best results for older adults, helping individuals improve their mental health.

#### 4.2.3. Measurement Tools

It was showed that physical exercise had a positive impact on the measurement tools of mental health in the Chinese older adults. The possible reasons for this result are as follows: first, the measurement dimensions were inconsistent between scales. Some scales only measure fixed variables, such as SAS and STAI, which measure anxiety. GDS and SDS, which measure depression, while SCL-90 and BFS measure somatization, fear, agitation, calmness, and other dimensions in addition to anxiety and depression. Second, the objects used in the scale were different. GDS was only applicable to the older adults, while other scales were applicable to the general person. The measurement dimensions between scales were inconsistent with the applicable objects, which might lead to some differences in the results of measurement tools. These results suggested that in the future, when choosing measurement tools, we should try to select scales developed for the older adults that fit the research needs. Compared with the other measurement tools, SCL-90 scale was the most widely used in mental health.

#### 4.2.4. Subject Older Adults Types

It was showed that physical exercise had a positive effect on the mental health of the subjects' older adults types. Different from other subjects, the older adults with hypertension suffer from both physical and psychological pressures, which jointly affect their mental health level. The main motivation for the older adults to participate in physical exercise is to enhance their physical health [39]. In the process of physical exercise, the older adults with hypertension will also bring this expectation into it, thus affecting the effect of physical exercise. This result is in line with the view of Maslow's hierarchy of needs theory. After the basic physiological needs were satisfied, the older adults with hypertension pursue higher levels of needs [40], and physical exercise just relieves the dual pressure of body and mind, achieving twice the result with half the effort.

### 4.3. Limitations

Due to the database limitations, the co-cited research was not analyzed. So, high-quality Chinese articles that have made important contributions in this field cannot be sorted out and cannot be compared with the articles in English. In the future, relevant research can further expand the scope of literature retrieval, research group, research content, and analyze current research hotspots and trends more comprehensively.

## 5. Conclusion

In this study, a meta-analysis was conducted to explore the effect of physical exercise on the mental health of the Chinese older adults. The results showed that: (1) physical exercise could improve the mental health, anxiety, and depression of the older adults to a certain extent; (2) The intervention effect of physical exercise on the mental health older adults was significantly moderated in the intervention types, intervention duration, intervention frequency, intervention time, measurement tools, and subject older adults types. Physical exercise had a positive effect on the mental health of the older adults, which was applicable to all older adults groups, but exercise rehabilitation was the most effective, and physical exercise had the best intervention effect on the older adults with hypertension. In order to achieve the intervention effect of improving mental health, it was recommended that the older adults do exercise a small number of times every day, 30 to 60 minutes each time, for 12 to 16 weeks to achieve the effect. In terms of measurement tools, future research should try to select scales developed for the older adults that fit the research needs.

## Figures and Tables

**Figure 1:** Article selection process.

**Figure 2:** Funnel Plot of effect of physical exercise on mental health of the older adults.

**Figure 3:** Funnel Plot of effect of physical exercise on anxiety of the older adults.

**Figure 4:** Funnel Plot of effect of physical exercise on depression of the older adults.

**Table 1:** PEDro scores of the included studies.

Study	Evaluation criterion											Scores
	1	2	3	4	5	6	7	8	9	10	11	
Xu [12]	1	1	1	1	0	0	0	1	1	1	0	6
Chen et al. [13]	1	1	1	1	0	0	1	1	1	1	0	7
Luo et al. [14]	1	1	1	0	0	0	0	1	1	1	0	5
Shen [15]	1	1	1	1	0	0	0	1	1	1	0	6
Sun and wang [16]	1	1	1	1	0	0	0	1	1	1	0	6
Zhang and Ma [8]	1	1	1	1	0	0	0	1	1	1	0	6
Zhao [17]	1	1	1	1	1	1	0	0	1	1	0	7
Zhao and Xu [18]	1	1	1	1	0	0	0	1	1	0	0	5
Ma et al. [19]	1	1	1	1	0	0	0	1	1	1	0	6
Gao [20]	1	1	1	1	1	1	0	1	1	1	0	8
Hou [21]	1	1	1	1	0	0	0	1	1	1	0	6
Ou [22]	1	1	1	1	0	0	0	1	1	1	0	6
Guan [23]	1	1	0	1	0	0	0	1	1	1	0	5
Sun [24]	1	1	1	1	0	0	0	1	1	1	0	6
Fan [25]	1	1	1	1	0	0	0	1	1	1	0	6

Note: 1. Eligibility criteria; 2. Randomization; 3. Allocation hidden; 4. Similar group baseline; 5. Blinding of all subjects; 6. Blinding of all therapists; 7. Blinding of all assessors; 8. Drops out <15%; 9. Intention to treat method; 10. Statistical between group; 11.print measures and measures of variability.

**Table 2:** Characteristics of studies included in the meta-analysis.

Author (year)	Intervention types	Intervention duration (min)	Intervention frequency (time)	Intervention time (week)	Measurement tools	Subject older adults types	Outcome variable
Xu [12]	Tai Chi	60	7	12	STAI	Healthy	Anxiety
Xu [12]	Dance	60	7	12	STAI	Healthy	Anxiety
Chen et al. [13]	Walk	20–30	5	16	SAS	Hypertension	Anxiety
Luo [14]	24-Form tai chi	60	3	24	SCL-90	Female	Anxiety, depression
Shen [15]	Square dance	60	4	12	SCL-90	Healthy	Anxiety, depression
Sun and wang [16]	Square dance	60	3	12	BFS	Healthy	Depression
Zhang and Ma [8]	Artery-relaxed scripture	45	7	8	SAS	Healthy	Anxiety
Zhao [17]	Fitness dance	90	3	12	GDS, SAS	Healthy	Anxiety, depression
Zhao and Xu [18]	Fitness dance	90	3	12	GDS	Healthy	Depression
Ma et al. [19]	Fitness walk	120	4–6	16	SCL-90	Empty nesters in rural areas	Anxiety, depression
Gao [20]	Qigong	60	5	24	SAS, SDS	Healthy	Anxiety, depression
Hou [21]	Tai Chi	30	7	24	SCL-90	Healthy	Anxiety, depression
Ou [22]	Tai Chi	60	3	24	SCL-90	Female	Anxiety, depression
Guan [23]	Square dance	50	3–4	12	SCL-90	Healthy	Anxiety, depression
Guan [23]	Five-animal exercises	50	3–4	12	SCL-90	Healthy	Anxiety, depression
Sun [24]	Exercise rehabilitation	30	7	48	SAS, SDS	Healthy	Anxiety, depression
Fan [25]	Exercise rehabilitation	20–30	3	48	SCL-90	Healthy	Anxiety, depression

**Table 3:** Studies included in the analyses.

Author (year)	Outcome variable	Intervention groups		Control groups	
		X1 ± SD1	n1	X2 ± SD2	n2
Xu (2005) [12]	Anxiety	21.75 ± 1.61	20	35.05 ± 5.27	14
Xu (2005) [12]	Anxiety	21.55 ± 5.96	18	35.05 ± 5.27	14
Chen et al. (2017) [13]	Anxiety	21.55 ± 5.96	18	35.05 ± 5.27	14
Luo (2008) [14]	Anxiety	23.02 ± 2.09	80	38.07 ± 3.74	80
Luo (2008) [14]	Depression	0.28 ± 0.31	40	0.45 ± 0.40	40
Shen (2016) [15]	Anxiety	0.22 ± 0.24	40	0.38 ± 0.41	40
Shen (2016) [15]	Depression	1.44 ± 0.44	20	1.67 ± 0.46	10
Sun and wang (2020) [16]	Depression	1.58 ± 0.38	20	1.79 ± 0.54	10
Zhang and Ma (2011) [8]	Anxiety	9.27 ± 3.22	40	13.24 ± 3.28	40
Zhao (2015) [17]	Anxiety	32.64 ± 8.84	21	44.62 ± 7.98	52
Zhao (2015) [17]	Depression	7.63 ± 2.81	30	10.77 ± 2.30	30
Zhao and Xu (2015) [18]	Depression	39.29 ± 4.29	30	46.54 ± 5.24	30
Ma et al. (2012) [19]	Anxiety	9.23 ± 2.62	30	10.00 ± 2.41	30
Ma et al. (2012) [19]	Depression	1.45 ± 0.59	60	1.52 ± 0.58	60
Gao (2016) [20]	Anxiety	1.37 ± 0.56	60	1.45 ± 0.61	60
Gao (2016) [20]	Depression	33.05 ± 6.49	149	36.73 ± 7021	37
Hou (2011) [21]	Anxiety	33.91 ± 6.21	149	36.99 ± 8.48	37
Hou (2011) [21]	Depression	0.23 ± 0.28	100	0.43 ± 0.44	100
Ou (2010) [22]	Anxiety	0.23 ± 0.27	100	0.35 ± 0.39	100
Ou (2010) [22]	Depression	0.28 ± 0.31	40	0.45 ± 0.40	40
Guan (2017) [23]	Anxiety	0.22 ± 0.24	40	0.38 ± 0.41	40
Guan (2017) [23]	Depression	1.33 ± 0.43	16	1.43 ± 0.47	16
Guan (2017) [23]	Anxiety	1.26 ± 0.24	16	1.36 ± 0.24	16
Guan (2017) [23]	Depression	1.20 ± 0.39	16	1.43 ± 0.47	16
Sun (2019) [24]	Anxiety	1.21 ± 0.27	16	1.36 ± 0.24	16
Sun (2019) [24]	Depression	46.01 ± 2.59	45	56.58 ± 3.15	45
Fan (2019) [25]	Anxiety	45.18 ± 2.37	45	56.35 ± 2.15	45
Fan (2019) [25]	Depression	12.64 ± 3.85	80	19.25 ± 4.34	80

**Table 4:** Publication bias and heterogeneity test.

Outcome variable	Number	Publication bias	Heterogeneity test		
		*Fail safe N*	Q	I^2^	*Tau-squared*
Mental health	28	3656	339.72	95.03	1.12
Anxiety	15	1268	331.86	95.78	1.42
Depression	13	606	206.60	94.19	0.91

**Table 5:** The effect of physical exercise on mental health of Chinese older adults.

Outcome variable	Number	SMD	LL	UL	Q	*P*
Mental health	28	−1.25	−1.66	−0.84	542.970	0.00
Anxiety	15	−1.45	−2.08	−0.83	331.86	0.00
Depression	13	−1.02	−1.56	−0.48	206.60	0.00

**Table 6:** The moderating effects of intervention methods on mental health of the older adults.

Outcome variable	Intervention methods	Number	SMD	LL	UL	*I* ^*2*^	*Q*	*P*
Mental health	Traditional exercise	12	−0.56	−0.68	−0.44	74.77	542.97	0.00
	Walk	3	−0.81	−1.04	0.57	99.99		
	Dance	9	−0.87	−1.08	−0.66	76.83		
	Exercise rehabilitation	4	−2.50	−2.74	−2.26	95.64		
Anxiety	Traditional exercise	7	−0.92	−1.39	−0.44	85.86	331.86	0.00
	Walk	2	−2.55	−7.28	2.19	99.42		
	Dance	4	−1.06	−2.02	0.10	85.79		
	Exercise rehabilitation	2	−2.62	−4.63	−0.61	96.39		
Depression	Traditional exercise	5	−0.49	−0.67	−0.32	0.00	206.60	0.00
	Walk	1	−0.12	−0.48	0.24	0.00		
	Dance	5	−0.73	−1.18	−0.27	66.74		
	Exercise rehabilitation	2	−3.77	−6.00	−1.55	95.60		

The effect of physical exercise duration on mental health, anxiety (*P* < 0.001), and depression (*P* < 0.001) of the older adults (*P* < 0.001) had a positive effect. Among them, the intervention effect on mental health (*d* = −2.51) and depression (*d* = −2.67) of the older adults when the single exercise duration less than 30 minutes is the largest, and the intervention effect on anxiety of the older adults was the largest when the exercise duration is 30–60 minutes (*d* = −1.21) (Table 7).

**Table 7:** The moderating effects of intervention duration on mental health of the older adults.

Outcome variable	Intervention duration	Number	SMD	LL	UL	*I* ^*2*^	*Q*	*P*
Mental health	<30 min	3	−2.51	−2.76	−2.26	97.62	542.97	0.00
	30–60 min	20	−0.75	−0.86	−0.64	92.26		
	>60 min	5	−0.46	−0.66	−2.26	97.62		
Anxiety	<30 min	2	−0.81	−2.16	0.54	98.80	331.86	0.00
	30–60 min	11	−1.21	−1.80	0.63	92.49		
	>60 min	2	−0.81	−2.16	0.54	93.72		
Depression	<30 min	1	−2.67	−3.09	−2.24	0.00	206.60	0.00
	30–60 min	9	−0.99	−1.60	−0.39	94.19		
	>60 min	3	−0.53	−1.16	0.11	81.88		

**Table 8:** The moderating effects of intervention frequency on mental health of the older adults.

Outcome variable	Intervention duration	Number	SMD	LL	UL	*I* ^*2*^	*Q*	*P*
Mental health	3–6	21	−0.85	−0.95	−0.74	93.91	542.97	0.00
	7	7	−1.08	−1.25	−0.91	97.14		
Anxiety	3–6	10	−1.07	−1.82	−0.32	95.86	331.86	0.00
	7	5	−2.28	−3.71	−0.85	96.44		
Depression	3–6	11	−0.75	−1.23	−0.27	90.74	206.60	0.00
	7	2	−2.72	−7.03	1.59	98.96		

The frequency of physical exercise on mental health, anxiety (*P* < 0.001), and depression (*P* < 0.001) of the older adults (*P* < 0.001) had a positive effect. Among them, the frequency of exercise 7 times a week on mental health (*d* = −1.08), anxiety (*d* = −2.28), and depression (*d* = −2.72) of the older adults which intervention effect was higher than 3–6 times a week (Table 8).

**Table 9:** The moderating effects of intervention time on mental health of the older adults.

Outcome variable	Intervention periods	Number	SMD	LL	UL	*I* ^*2*^	*Q*	*P*
Mental health	<12	1	−1.46	−2.01	−0.90	0.00	542.97	0.00
	12–16	15	−0.87	−1.01	−0.72	94.58		
	>16	12	−0.91	−1.03	−0.80	96.08		
Anxiety	<12	1	−1.46	−2.01	−0.90	0.00	331.86	0.00
	12–16	8	−1.70	−2.98	−0.43	96.77		
	>16	6	−1.15	−1.89	−0.42	95.19		
Depression	12–16	7	−0.59	−0.98	−0.21	70.90	206.60	0.00
	>16	6	−1.54	−2.54	−0.53	97.15		

**Table 10:** The moderating effects of physical exercise on the effect of measurement tools of mental health in the older adults.

Outcome variable	Measurement tools	Number	SMD	LL	UL	*I* ^*2*^	*Q*	*P*
Mental health	GDS	2	−0.73	−1.10	0.35	82.57	542.97	0.00
	SAS	5	−1.84	−2.08	−1.61	97.71		
	SCL−90	16	−0.63	−0.74	−0.53	89.48		
	SDS	2	−1.18	−1.51	−0.84	98.93		
	STAI	2	−2.91	−3.62	−2.21	69.66		
	BFS	1	−1.22	−1.70	−0.74	0.00		
Anxiety	SAS	5	−2.42	−4.02	−0.83	97.71	331.86	0.00
	SCL−90	8	−0.53	−0.93	−0.13	83.81		
	STAI	2	−3.01	−4.31	−1.70	69.66		
Depression	GDS	2	−0.76	−1.66	0.14	82.57	206.60	0.00
	SCL−90	8	−0.70	−1.30	−0.09	92.84		
	SDS	2	−2.68	−7.07	1.71	98.93		
	STAI	1	−2.38	−3.29	−1.47	0.00	STAI	

**Table 11:** The moderating effects of physical exercise on the mental health of subject older adults types.

Outcome variable	Subject elderly types	Number	SMD	LL	UL	*I* ^*2*^	*Q*	*P*
Mental health	Healthy	21	−1.03	−1.14	−0.93	93.84	542.97	0.00
	Female	4	−0.46	−0.69	−0.24	0.00		
	Hypertension	1	−4.97	−5.59	−4.34	0.00		
	Empty nesters in rural areas	2	−0.13	−0.38	0.13	0.00		
Anxiety	Healthy	11	−1.43	−2.03	−0.82	93.07	331.86	0.00
	Female	2	−0.48	−0.79	−0.16	0.00		
	Hypertension	1	−4.97	−5.59	−4.34	0.00		
	Empty nesters in rural areas	1	−0.14	−0.50	0.22	0.00		
Depression	Healthy	10	−1.24	−1.94	−0.54	95.00	206.60	0.00
	Female	2	−0.45	−0.77	−0.14	0.00		
	Empty nesters in rural areas	1	−0.12	−0.48	0.24	0.00		

## Data Availability

The datasets used and/or analyzed during the current study are available from the corresponding author on reasonable request.
